# Diagnosis of Neural Activity among Abnormal Brain Regions in Patients with Major Depressive Disorder by Magnetic Resonance Imaging Features

**DOI:** 10.1155/2022/3044010

**Published:** 2022-06-28

**Authors:** Weicheng Wang, Shuang Jia, Qionghui Zhao, Lin Yang

**Affiliations:** ^1^Department of Radiology, Affiliated Hospital of North Sichuan Medical College, Nanchong 637000, China; ^2^Department of Radiology, Nanchong Hospital of Traditional Chinese Medicine, Nanchong 637000, China

## Abstract

In order to explore the diagnostic value of magnetic resonance imaging (MRI) for neural activity among abnormal brain regions in patients with major depressive disorder (MDD), thirty patients with MDD (observation group) were selected for comparison with 30 healthy people without MDD (control group). The included subjects were examined by MRI to compare the MRI features and were analyzed for regional homogeneity (ReHo) and amplitude low-frequency fluctuations (ALFF). The results showed that compared with the control group, the brain regions with increased ReHo and ALFF in the observation group were medial frontal gyrus (right), middle temporal lobe (left), inferior parietal lobe (left), and posterior cerebellar lobe (right); the brain region with increased ReHo and ALFF in the observation group was the middle temporal gyrus (right). Compared with the control group, there were significant differences in ReHo and ALFF in the observation group. It was found that the brain function of patients with MDD was abnormal compared with that of the normal subjects, and the brain network activity was also abnormal. MRI features can be used to explore abnormal brain regions in patients with MDD and have positive guiding value.

## 1. Introduction

Depressive disorder is a dangerous condition that affects the patient's physical and mental status. According to the estimation of the WHO, the suicide rate of depressive disorder is 12%-14%, and its disability is second only to chronic obstructive pulmonary disease [1]. Major depressive disorder (MDD) is a disease that severely affects patients' mood, and patients are in a poor state of depression and lack of interest [2]. The lifetime prevalence of MDD ranges from 10% to 25% in women and from 5% to 12% in men. The incidence is significantly higher in the female population than in the male population [3]. More than half of suicides suffer from MDD or other mood disorders, so the treatment and prevention of MDD is important [4]. The incidence of MDD is very high, and recurrence is highly likely after treatment. Patients often have suicidal thoughts and are at high risk, placing a high burden of disease on patients and their families [5]. MDD is a mental illness that seriously endangers human health and seriously affects the quality of life of patients, and patients are prone to injury during the onset of the disease and have a high rate of disability. Therefore, it poses a great threat to the patient's normal life.

Positron emission tomography (PET) and single-photon emission computed tomography (SPECT) are commonly adopted to explore depressive disorder [6]. In recent years, functional magnetic resonance imaging (fMRI) has been widely used. With its high temporal and spatial resolution, convenient operation, no exposure to radioactive active substances, and no trauma, it has become a commonly used research method, with the unique value in the exploration of depression [7]. The fMRI is a new examination technology. Compared with other examination methods, it has unique advantages and is widely applied in brain neuroscience and psychological cognition, with good results [8]. The objective of fMRI is mainly to explore brain activation. Under specific conditions, the neural activity in the brain and various brain regions is analyzed. Moreover, the control state in task state and no task state is subtracted to obtain a result that is the brain activation signal. The brain activation signal reflects the relevant activities of task-related brain nerves [9]. In functional MRI experiments, the normal control group is generally in a resting state. The functional brain activity of the observation group is obtained by subtracting the resting state from the task state [10]. The resting state is a stable and quiet state, which means that the experiment is performed when patients are in a state of relaxation, without external interference. The signal receiving of this method is weak, so there are certain requirements for images and data processing of magnetic resonance instruments. Currently, there are many data analysis methods for resting state, such as brain functional connection, regional consistency, and independent component analysis. The various methods have different perspectives on data processing, all of which have certain effects. The fMRI has an important adoption value in the study of MDD [11].

The neural activity among the abnormal brain regions of patients with MDD was investigated based on the MRI features. The research objects received the MRI examination, and the images were processed and analyzed. The regional homogeneity (ReHo) analysis and amplitude low-frequency fluctuation (ALFF) analysis were performed, and the MNI by the *Montreal Neurological Institute* of the ReHo and the ALFF differences in brain regions were counted. The adoption effect of MRI in the diagnosis and prediction of patients with MDD was analyzed. It was hoped to provide clinical guidance for the image processing of MRI and analysis of patients with MDD and provide a reference for the diagnosis and prediction of patients with MDD.

## 2. Materials and Methods

### 2.1. Research Objects

Thirty patients with MDD admitted from March 2018 to March 2021 (observation group) were selected for comparison with 30 healthy people without MDD (control group). MRI was performed on the included subjects, and the MRI characteristics were compared. This study was approved by the ethics committee of hospital and informed consents were obtained from subjects.

For the observation group, the inclusion criteria were as follows: (I) patients with complete medical records and imaging data; (II) patients whose ages ranged from 18 to 55 years old; (III) patients who met the diagnostic criteria of unipolar depression in the Chinese *Diagnostic and Classification Criteria of Mental Disorders* (CCMD--3) and the diagnostic criteria of MDD in the American *Diagnostic and Statistical Manual of Mental Disorders* (DSM-IV); (IV) patients with the 24 Hamilton depression scale (HAMD) scores ≥35; and (V) patients who signed the informed consent. The exclusion criteria were as follows: (I) patients with diseases of vital organs; (II) patients who suffered from central nervous system diseases, endocrine system diseases, and other serious physical diseases; (III) patients in pregnancy or lactation; and (IV) patients who were unwilling to participate in the experiment.

For the control group, the inclusion criteria were as follows: (I) patients with complete imaging data, (II) patients with the age from18 to 55 years old, and (III) patients with the HAMD scores ≤8. The exclusion criteria were as follows: (I) patients with MRI contraindications; (II) patients who abused alcohol, drugs, or other psychoactive substances; (III) patients in pregnancy or lactation; (IV) patients with mental disorders; and (V) patients with diseases of other vital organs.

### 2.2. MRI Examination

1.5 T magnetic resonance scanner was used for inspection, and channel parallel instrument collector coil was used for signal reception. During the examination, the patient remained supine position and wore a dedicated nonmagnetic earphone. The scan process was as follows. Conventional three-plane localization and the gradient echo-planar imaging (GRE-EPI) sequence recalled were adopted. With the anterior and posterior wiring as scan baseline, the oblique axial scanning was implemented, ranging from the patient's calvarium to the foramen magnum. The parameters are as follows: time of repetition (TR) = 2000 ms, time of echo (TE) = 30 ms, field of view (FOV) = 240 mm × 240 mm, matrix = 64 × 64, flip angle = 90°, scanning = 30 layers continuously, layer thickness = 5 mm, and layer interval = 0 mm.

### 2.3. Image Processing and Analysis

#### 2.3.1. Data Preprocessing

DPARSF toolbox was employed for the preprocessing of the original images. To rule out the effect that patients' inadaptation of the scanning instrument environment, noise, and longitudinal relaxation of magnetization did not reach the steady state on the results, the data of the first 10 points were eliminated. The content was the data of the following 190 time points, which guided the patients for the correction of head movement. The translational motion of all included data in all directions (*X*, *Y*, and *Z*) was less than 1.5 mm, with the rotation angle less than 1.5° to reduce the interference of the signal caused by the noise because of the head movement in the scanning process. For time point correction, there was a time difference in acquisition among 30 layers of image signals at each time point, so the time differences among the layers are needed to be corrected. According to the time modulation effect of the hemodynamic function on the functional images of each layer, the images collected at different time points were corrected at the same time point. There were anatomical differences in the brains of the research objects, so different images are needed to be spatially standardized, which meant that they were transformed into standardized images with the same size and orientation. Meanwhile, they were in the same standard three-dimensional space and the same coordinate system. In the process of standardization, a standard brain structure image template was required. The MNI template proposed by the *Montreal Neurological Institute* was adopted, and the images were standardized onto the standard EPI template of the statistical parametric mapping (SPM5). Then, the brain images with a voxel size of 3 mm × 3 mm × 3 mm were generated. Finally, the standardized image was filtered (Figure 1).

#### 2.3.2. ReHo Analysis

The local consistency referred to the synchronization of the time series of each voxel and its adjacent voxel in the whole brain. The Kendall coefficient of concordance (KCC) was used as an index to measure the consistency of time series changes, which could effectively reflect the similarity degree among time series of different voxels in a functional region. The KCC was assigned to the voxel, with a value from 0 to 1. Each voxel had a ReHo value, and a ReHo image of the whole brain was formed. Equation (1) shows how the KCC value was calculated. In Equation (1), *W* represented the total KCC value of the selected voxels, *Ri* represented the sum of the rank of the *i*th time point, *R* represented the mean value of *Ri*, *n* represented the times of total rank, and *K* represented the number of time series in the measuring cell. After the KCC of the whole brain was calculated, the image was smoothed by the 4 mm full-width half-height filtering.

(1) $$\begin{array}{c} W=\frac{\sum {\left(R_{i}\right)}^{2}-n{\left(\bar{R}\right)}^{2}}{\left(1/12\right)K^{2}\left(n^{3}-n\right)}. \end{array}$$

#### 2.3.3. ALFF Analysis

The ALFF value reflected the level of spontaneous activity of each voxel in the resting state from the perspective of energy. The software was employed for the calculation of the mean value of amplitude in a frequency band at all frequency points, and the ALFF analysis was performed for the graph of each individual that was obtained after smoothing.

### 2.4. Observation Indexes

The general data, including gender, age, years of education, and HAMD score, was compared between the two groups. HAMD scale was adopted to assess the severity of depression. The higher the score was, the more severe the severity was. When the score was >14, it was depression.

The ReHo value, ALFF value, and brain region image of the two groups were analyzed.

### 2.5. Statistical Methods

The data was used to record and summarize. SPSS 20.0 was used for data statistics and analysis. Mean ± standard deviation$\left(\overset{¯}{x}\pm s\right)$ indicated measurement data, and *t*-test was used. Percentage (%) was the expression of count data, and *χ*^2^ test was adopted. *P* < 0.05 was considered statistically significant.

## 3. Results

### 3.1. Comparison of General Data

Table 1 shows the comparison of general data between the two groups. The male-to-female ratio was 11/19 for the control group, and that was 12/18 for the observation group. The average age of patients in the control group was 31.78 ± 8.72 years old, and that in the observation group was 31.27 ± 8.66 years old. The year of education of the patients in the control group was 12.78 ± 2.57 years, and that in the observation group was 12.65 ± 2.78 years. The HAMD score of the control group was 3.17 ± 1.38, and that of the observation group was 33.68 ± 1.52. There were statistically insignificant differences in general data between the two groups (*P* > 0.05), with comparability.

### 3.2. MNI Comparison of ReHo Differences in Brain Regions

Figure 2 shows the brain regions with increased ReHo in the observation group compared with the normal control group, and Figure 3 shows that with decreased ReHo. Compared with the normal control group, the brain regions with increased ReHo in the observation group were the medial frontal gyrus (right), anterior central gyrus (left), superior temporal gyrus (right), middle temporal gyrus (left), angular gyrus (right), inferior parietal lobule (left), insula (left), thalamus (left), and posterior lobe of the cerebellum (right). The brain regions with decreased ReHo were the superior frontal gyrus of the orbit (right), orbital middle frontal gyrus (left), middle temporal gyrus (right), anterior cingulate gyrus (right), posterior cingulate gyrus, and inferior parietal lobule (right).

### 3.3. The ReHo Differences in Brain Region Images

Figure 4 shows the ReHo differences in brain regions in the observation group compared with the control group (red indicated increased activation, and blue indicated decreased activation). The ReHo of the superior frontal gyrus of the orbit (right) and orbital middle frontal gyrus (left) in the observation group decreased markedly compared with the control group. The ReHo of the anterior central gyrus (left), superior temporal gyrus (right), and middle temporal gyrus (left) in the observation group increased compared with the control group.

### 3.4. MNI Comparison of ALFF Differences in Brain Regions

Figure 5 shows the brain regions with the increased ALFF in the observation group compared with the normal control group, and Figure 6 shows that with the decreased ALFF. Compared with the normal control group, the brain regions with the increased ALFF in the observation group mainly included the superior frontal gyrus (left), inferior frontal gyrus (right), medial frontal gyrus (right), middle temporal gyrus (left), inferior parietal lobule (left), thalamus (left), posterior lobe of the cerebellum (left), and posterior lobe of the cerebellum (right). Additionally, the brain regions with the decreased ALFF in the observation group included the parahippocampal gyrus (right), middle temporal gyrus (right), lingual gyrus (right), inferior parietal lobule (right), middle frontal gyrus (right), and posterior central gyrus (right).

### 3.5. The ALFF Differences in Brain Region Images

Figure 7 shows the ALFF differences in brain regions in the observation group compared with the control group (red presented the increased activation, and blue presented the decreased activation). Compared with the control group, the ALFF of the middle temporal gyrus (right) and other regions in the observation group decreased obviously, while that of the inferior frontal gyrus (right) and other regions increased.

## 4. Discussion

In recent years, the incidence of depression has been increasing and severely affects human health and quality of life [12]. Depression has some physical and psychological impact on patients, affecting their normal work and life as well as their psychological state, thus making them depressed and losing interest in life [13, 14]. MDD severely affects the patients themselves and their families. Negative emotions have a negative impact on patients, and patients may lose their enthusiasm, immerse themselves in negative emotions, and fail to live a normal life [15, 16]. With the continuous progress of science and technology, imaging is also developing rapidly. MRI technology has now become a routine examination, superior to other examination methods, and is the diagnostic technique of choice for many diseases. A noninvasive examination method can significantly reduce the discomfort of patients with high safety. Multimodality MRI examination mainly includes brain fMRI, high-resolution structural imaging, and diffusion tensor imaging (DTI). fMRI of the brain has the advantage of MRI itself and provides new ideas and methods for exploring the working mechanisms and rules of the brain, which has some clinical value in reflecting the relationship between the functional connectivity and anatomical connectivity of brain networks [17, 18].

According to some related studies of fMRI, depressed patients have abnormal brain structure and functional status, and in addition, abnormal brain function at specific sites can be reversed after some specific drug treatment [19]. In fMRI, brain function is analyzed by analyzing changes in cerebral hemodynamics to explore the mechanisms and characteristics of neural activity and functional connectivity in brain regions [20, 21]. It has been found that ReHo values in the median cingulate, posterior central gyrus (right), and anterior central gyrus were significantly lower during the first episode (FE) in MDD patients compared with healthy controls [22]. Liu et al. [23] explored the expression recognition and locomotor activity characteristics of the resting brain in MDD patients. It was found that ReHo values were decreased in the left parascapular gyrus, left thalamus, right putamen, left putamen, and right angular gyrus and increased in the left superior frontal gyrus, left middle temporal gyrus, left medial superior frontal gyrus, and right medial superior frontal gyrus in the MDD patients compared with healthy controls. It analyzed neural activity in abnormal regions of the brain in MDD patients and explored the effect of MRI in the diagnosis and prediction of patients with MDD. The novelty of the experiment is that ReHo analysis and ALFF analysis are performed on the MRI images of the study subjects, and MNI in the brain regions with differential ReHo and ALFF is counted. The results showed that compared with the normal control group, the brain regions with increased ReHo in the observation group were medial frontal gyrus (right), anterior central gyrus (left), superior temporal gyrus (right), middle temporal gyrus (left), angular gyrus (right), inferior parietal lobe (left), insular lobe (left), thalamus (left), and posterior cerebellar lobe (right). Brain regions with decreased ReHo were the superior orbital frontal gyrus (right), middle orbital frontal gyrus (left), middle temporal gyrus (right), anterior cingulate (right), posterior cingulate, and inferior lobe (right). In addition, compared with the normal control group, the brain regions with increased ALFF in the observation group were mainly superior frontal gyrus (left), inferior frontal lobe (right), medial frontal gyrus (right), middle temporal lobe (left), inferior parietal lobe (left), thalamus (left), posterior cerebellar lobe (left), and posterior cerebellar lobe (right). The brain regions with decreased ALFF in the observation group included the parahippocampal gyrus (right), middle temporal gyrus (right), lingual gyrus (right), inferior parietal lobe (right), middle frontal lobe (right), and posterior central gyrus (right). This may be due to altered cerebral hemodynamics in patients with MDD, abnormal brain function compared to normal subjects, and abnormal brain network activity.

## 5. Conclusion

The exploration of neural activities in abnormal brain regions of patients with MDD under the imaging features of MRI had the guiding significance. It could provide the reference for the diagnosis and prediction of MDD, which was worthy of clinical adoption. The deficiency of this experiment is that the sample size is small, which requires further research and verification.

## Figures and Tables

**Figure 1:** Flow chart of data preprocessing.

**Figure 2:** Brain regions with increased ReHo in observation group compared with control group. *X*, *Y*, and *Z* are MNI coordinate axes (mm).

**Figure 3:** Brain areas with decreased ReHo in the observation group compared with control group. *X*, *Y*, and *Z* are MNI coordinate axes (mm).

**Figure 4:** Brain regions with ReHo difference compared with control group: (a) transverse plane; (b) sagittal plane; (c) coronal plane.

**Figure 5:** Brain regions with increased ALFF in the observation group compared with control group. *X*, *Y*, and *Z* are MNI coordinate axes (mm).

**Figure 6:** Brain regions with decreased ALFF in the observation group compared with control group. *X*, *Y*, and *Z* are MNI coordinate axes (mm).

**Figure 7:** Brain regions with ALFF difference compared with control group: (a) transverse plane; (b) sagittal plane; (c) coronal plane.

**Table 1:** Comparison of the general data between the two groups.

	Male/female	Age	Years of education	HAMD
Control group	11/19	31.78 ± 8.72	12.78 ± 2.57	3.17 ± 1.38
Observation group	12/18	31.27 ± 8.66	12.65 ± 2.78	33.68 ± 1.52

## Data Availability

The data used to support the findings of this study are available from the corresponding author upon request.
